The article "In vivo and in vitro effects of heme oxygenase-1 silencing on the survival of acute myelocytic leukemia-M2 cells" was retracted in 2025. Reasons: duplicated data; overlap with earlier publications; unreliable data; concerns about the data.

# *In vivo* and *in vitro* effects of heme oxygenase-1 silencing on the survival of acute myelocytic leukemia-M2 cells

**DOI:** 10.3892/etm.2015.2209

**Published:** 2015-01-23

**Authors:** SIXI WEI, YATING WANG, QIXIANG CHAI, QIN FANG, YAMING ZHANG, JISHI WANG

**Affiliations:** 1 Department of Hematology, The Affiliated Hospital of Guiyang Medical College, Guiyang, Guizhou 550004, P.R. China; 2 Hematopoietic Stem Cell Transplantation Center of Guizhou Province, The Affiliated Hospital of Guiyang Medical College, Guiyang, Guizhou 550004, P.R. China; 3 Department of Clinical Biochemistry, The Affiliated Hospital of Guiyang Medical College, Guiyang, Guizhou 550004, P.R. China; 4 Department of Pharmacy, The Affiliated Hospital of Guiyang Medical College, Guiyang, Guizhou 550004, P.R. China

**Keywords:** heme oxygenase-1, proliferation, apoptosis, infiltration

## Abstract

The aim of this study was to investigate the *in vivo* and *in vitro* effects of targeted heme oxygenase-1 (HO-1) silencing on the proliferation and apoptosis of human acute myelocytic leukemia (AML)-M2 cells. Bone marrow mononuclear cells (BMMNCs) were infected by pRNAi-siHO-1-GFP. The viability of the BMMNCs was determined by cell counting kit-8 (CCK-8) assay following daunorubicin (DNR) treatment. The apoptotic rate was detected by flow cytometry. The expression levels of HO-1 and apoptosis-related genes were detected by quantitative polymerase chain reaction (qPCR) and western blot analysis. An AML-M2 xenograft mouse model was established. The tumor formation outcomes and survival were observed. The leukocyte and platelet counts and hemoglobin levels were monitored, and the copy numbers of AML1/ETO fusion gene were detected by qPCR. pRNAi-siHO-1-GFP silenced the expression of HO-1. DNR inhibited cell viability in a time- and dose-dependent manner. The survival rate of the cells was significantly reduced by infection with pRNAi-siHO-1-GFP. HO-1 expression in the BMMNCs infected with pRNAi-siHO-1-GFP was downregulated, whereas caspase-3, -8 and -9 expression was upregulated compared with that in control BMMNCs. Kasumi-1 cells were successfully inoculated into nude mice. The rats inoculated with pRNAi-siHO-1-GFP-transfected Kasumi-1 cells succumbed to tumors more slowly and survived longer than those inoculated with untransfected Kasumi-1 cells. Furthermore, the leukocyte and platelet counts and hemoglobin levels were higher and the copy numbers of AML1/ETO fusion gene were lower in the former group. HO-1 gene silencing may promote the apoptosis of human M2 leukemic cells by inhibiting a caspase-dependent apoptotic pathway. Targeted silencing of HO-1 is able to inhibit the proliferation and infiltration of leukemic cells in nude mice and thus prolong their survival. The findings provide valuable experimental evidence for the molecular targeted therapy of M2 leukemia.

## Introduction

Acute myelocytic leukemia (AML), which results from the malignant cloning of myeloid progenitor cells in the hematopoietic system, is mainly treated by chemotherapy and hematopoietic stem cell transplantation currently. However, the disease-free and overall survival rates remain low due to the toxicity and high recurrence rate of chemotherapy, strict selection of transplant donors and recipients and severe complications (1,2). Therefore, the identification of eligible targets for AML therapy is now of global interest.

Heme oxygenase-1 (HO-1), also known as heat shock protein (HSP) 32, is located on human chromosome 22q12 while being highly conserved and its expression can be induced by various stimulatory factors (3). HO-1 affects the growth of solid tumors in many aspects, and it is expressed at higher levels in cancer cells, for example, in renal cell carcinoma, squamous cell carcinoma, brain cancer, Kaposi’s sarcoma, lung cancer, pancreatic cancer and melanoma, than in normal tissues (4–6). In many types of tumors, HO-1 protects cells from apoptosis, promotes cell proliferation and enhances tumor invasion (7–9). Furthermore, the HO-1 level is associated with the occurrence and development of hematological diseases. When highly expressed, it protects leukemia cells from chemotherapy drugs, reduces apoptosis and enhances drug resistance (11–13). Our group has been studying the association between HO-1 and leukemia. It has been found that the inhibition of HO-1 expression can increase the sensitivity of AML mononuclear cells to chemotherapy (14). In addition, HO-1 has been demonstrated to be involved in the regulation of the survival and apoptosis of chronic myeloid leukemia (CML) cells and to be associated with CML disease progression and drug resistance (15–17). Since HO-1 is significantly highly expressed in patients with leukemia compared with normal subjects, downregulating HO-1 expression may provide new protocols for the treatment of leukemia. Nevertheless, little has been reported about the effects of downregulated HO-1 expression on the proliferation and apoptosis of AML cells. In particular, relevant *in vivo* and *in vitro* studies remain scarce.

Therefore, HO-1 expression in human AML-M2 bone marrow mononuclear cells (BMMNCs) was silenced through infection using a lentiviral vector with HO-1 small interfering RNA (siRNA). The effect of silenced HO-1 gene expression on the proliferation and apoptosis of mononuclear cells was evaluated *in vitro*. In addition, an AML1/ETO-positive Kasumi-1 cell-inoculated AML-M2 xenograft mouse model was established to explore the effects of targeted silencing of HO-1 expression by the green fluorescent protein (GFP)-expressing plasmid pRNAi-siHO-1-GFP on the *in vivo* proliferation and infiltration of leukemic cells. The results should provide experimental evidence for verifying the role of HO-1 regulation in the treatment of AML-M2.

## Materials and methods

### Samples

Bone marrow/peripheral blood mononuclear cells from AML-M2 patients and the AML-M2 Kasumi-1 cell line (The Center Laboratory of the Hematopoietic Stem Cell Transplantation Center of Guizhou Province, Guiyang, China) were used as samples.

### Testing of HO-1 expression in AML-M2 patients by reverse transcription-polymerase chain reaction (RT-PCR)

Twenty peripheral blood samples were collected from AML-M2 patients and another 20 were collected from normal subjects. This study was conducted in accordance with the Declaration of Helsinki and with approval from the Ethics Committee of Guiyang Medical College (Guiyang, China). Written informed consent was obtained from all participants. Mononuclear cells were separated using Ficoll-lymphocyte separation medium (Beyotime Institute of Biotechnology, Nanjing, China). Total RNA was isolated and purified from cells using the RNeasy kit (Qiagen, Hilden, Germany). For RT-PCR analysis, 2,000 ng of RNA was reverse transcribed into cDNA with the Omniscript Reverse Transcription kit (Qiagen) in 20 μl of reaction volume. Amplification was performed by Veriti^®^ 96-Well Fast Thermal cycler (Applied Biosystems, Foster City, CA, USA). An equal amount of mRNA was loaded and run on a 5% SDS-PAGE gel. Details of the primers (HO-1^RT^) are listed in Table I. Conditions for the RT-PCR reaction were as follows: 40 sec at 53°C and 58°C, 6 min at 94°C, followed by 30 cycles, each consisting of 40 sec at 94°C and 50 sec at 72°C. The relative expression of HO-1 was demonstrated by the ratio of the gray scale between HO-1 and GAPDH.

### Conventional culture of Kasumi-1 cells

The Kasumi-1 cells were maintained in Roswell Park Memorial Institute-1640 (RPMI-1640; Hangzhou Sijiqing Biological Engineering Materials Co., Ltd., Hangzhou, China) culture medium containing 10% fetal bovine serum (Hangzhou Sijiqing Biological Engineering Materials Co., Ltd.) at 37°C in saturated humid air in a 5% CO_2_ incubator. The cells were passaged every 3–4 days when the culture medium was also refreshed, and they were inoculated at the density of 1×10^5^/ml.

### Preparation and culture of BMMNCs

Ten AML-M2 patients (five males and five females) enrolled in the Hematopoietic Stem Cell Transplantation Center of Guizhou Province (Guiyang, China) from March 2010 to March 2012 were selected. Under sterile conditions, 2 ml bone marrow blood was drawn, into which was added 2 ml Ficoll-lymphocyte separation medium (relative density: 1.007). After the sample was subjected to horizontal centrifugation at 229 × g for 10 min, the mononuclear cell layer was collected, washed and precipitated as BMMNCs. The rate of viable cells was >90%, as indicated by staining with 0.4% trypan blue. The separated BMMNCs were inoculated in RPMI-1640 culture medium containing 20% fetal bovine serum, 100 μg/ml penicillin and 100 μg/ml streptomycin, and were cultured and passaged at 37°C in saturated humid air in a 5% CO_2_ incubator.

### Infection of BMMNCs with the recombinant lentivirus pRNAi-siHO-1-GFP

The siRNA sequence for the coding sequence of HO-1 mRNA was designed as follows: 5′-AAGCUUUCUGGUGGCGACAGU-3′. HO-1-targeted siRNA, pRNAi-siHO-1-GFP and pRNAi-GFP were packaged and produced by Biomics Biotechnologies Co., Ltd. (Nantong, China). Kasumi-1 cells and BMMNCs in the logarithmic growth phase were inoculated at the concentration of 1×10^6^ cells/well in 6-well plates following overnight culture and were subsequently transfected with pRNAi-GFP (with/without siHO-1) at multiplicities of infection of 8 in serum-free medium. Polybrene (5 μg/ml; Sigma-Aldrich, St. Louis, MO, USA) was added to improve transfection efficiency as an enhancing reagent. After 10 h, the medium was changed for complete medium and the cells without intervention were used as the blank control group The experimental group was further divided into a normal BMMNC group (BMMNC), a pRNAi-siHO-1-GFP-infected BMMNC group (pRNAi-siHO-1-BMMNC) and a GFP empty vector-infected BMMNC group (pRNAi-GFP-BMMNC). The fluorescence intensity of GFP was observed under a fluorescence microscope (BX51; Olympus Corporation, Tokyo, Japan).

### Cell viability assay

Three cell groups in the logarithmic growth phase were inoculated onto 96-well plates at a density of 4×10^5^/ml. After 12 h of culture, different concentrations of DNR (Sigma-Aldrich; 0, 2.5, 5, 7.5, 10 and 12.5 μg/ml) were added to the wells. The inhibitory effects of DNR were determined using the cell counting kit (CCK-8) assay (Beyotime Institute of Biotechnology).

### Detection of cell apoptosis

Apoptotic cells were analyzed by flow cytometry with propidium iodide (PI) staining (BD Biosciences, San Jose, CA, USA). In brief, cells of the three groups in the logarithmic growth phase were inoculated onto 6-well plates at a final density of 1×10^5^/ml. After 12 h of culture, the cells were treated with different concentrations of DNR (0, 5 and 10 μg/ml) for 48 h. Then, 1×10^5^ cells were collected and washed twice with pre-cooled 1X phosphate-buffered saline (PBS). After suspending the cells by adding 500 μl 1X binding buffer (Solarbio Science & Technology Co., Ltd., Beijing, China) to each tube, they were further stained by adding 5 μl Annexin V-FITC solution (Beyotime Institute of Biotechnology) and 5 μl PI solution sequentially. Subsequently, the solution was allowed to react for 15 min in the dark at room temperature, and cell apoptosis was detected by flow cytometry using the BD FACSCalibur^™^ flow cytometer with BD CellQuest^™^ software (BD Biosciences, Franklin Lakes, NJ, USA) within 1 h.

### Quantitative PCR (qPCR)

pRNAi-siHO-1-BMMNCs in the logarithmic growth phase were inoculated onto 6-well plates at the final density of 1×10^6^/ml. Various concentrations of DNR (0, 5, 7.5, 10 and 12.5 μg/ml) were added and the cells were cultured for 48 h. RT-PCR was performed using an RT-PCR thermocycler (Applied Biosystems) and quantified using SYBR^®^ Green PCR Master mix (Applied Biosystems) using 1 μl cDNA in a final reaction volume of 20 μl. The names, sequences and amplified fragments of the primers (Applied Biosystems) are summarized in Table I. The PCR reactions were cycled 45 times after initial denaturation (94°C for 1 min) with the following parameters: denaturation at 94°C for 10 sec; annealing at 58°C for 15 sec (caspase-3, caspase-8 and GAPDH), at 60°C for 10 sec (caspase-9), or at 64°C for 10 sec (HO-1), and extension at 72°C for 15 sec. GAPDH was used as the internal control. SDS 2.2.1 software (Applied Biosystems) was used to perform relative quantification of the target genes using the 2-^ΔΔ^Ct method.

### Western blotting

BMMNCs and pRNAi-siHO-1-BMMNCs in the logarithmic growth phase were inoculated onto 6-well plates at a final density of 1×10^6^/ml. Following the addition of 5 μg/ml DNR for 48 h, the cells were washed in PBS, collected, and then lysed in radioimmunoprecipitation assay buffer (50 mmol/l Tris-HCl; 150 mmol/l NaCl; 0.1% SDS; 0.5% Na-deoxycholate and 1% NP-40) containing proteinase inhibitor cocktail and phosphatase inhibitor cocktail (Roche Applied Science, Indianapolis, IN, USA). The lysate was centrifuged at 10,000 × g at 41°C for 10 min. The supernatant (50–100 mg protein) was fractioned by SDS-PAGE using 10% gels and was transferred electrophoretically to Hybond-enhanced chemiluminescence membranes (GE Healthcare Life Sciences, Piscataway, NJ, USA). The membrane was blocked with blocking buffer (Li-Cor Biosciences, Lincoln, NE, USA) at room temperature for 1 h and then incubated with the monoclonal primary antibody [rabbit anti-human HO-1 (1:500), rabbit anti-human caspase-9 (1:500), mouse anti-human caspase-3 (1:500), mouse anti-human caspase-8 (1:500) and mouse anti-human β-actin (1:1,000); Cell Signaling Technology, Inc., Danvers, MA, USA] at 4°C overnight. After being washed with PBS with 0.1% Tween 20 (PBST), the membrane was incubated with horseradish peroxidase-labeled anti-rabbit IgG (1:1,000; Santa Cruz Biotechnology, Santa Cruz, CA, USA) and anti-mouse IgG (1:1,000; Santa Cruz Biotechnology) for 1 h at room temperature. The membrane was washed with PBST again and detected by electrochemiluminescence (Beyotime Institute of Biotechnology). By using β-actin expression as the internal reference, the protein expression levels were calculated using ImageJ software, V4.0 (National Institutes of Health, Bethesda, MD, USA).

### Inoculation of nude mice with AML1/ETO-positive Kasumi-1 cells

Under sterile conditions, 40 nude mice aged 5–6 weeks with weights of 18–22 g were selected (Guiyang Medical College). The numbers of male and female mice were equal. This study was carried out in strict accordance with the recommendations in the Guide for the Care and Use of Laboratory Animals of the National Institutes of Health (The National Academy Of Sciences, Washington D.C, 1996). The animal use protocol was reviewed and approved by the Institutional Animal Care and Use Committee (IACUC) of Guiyang Medical College.

Kasumi-1 cells in the logarithmic growth phase were collected and adjusted to a density of 1,000×10^4^/ml. The mice were divided into four groups (n=10 per group). The blank group was left untreated, the normal saline group was subcutaneously injected with normal saline, the Kasumi group was inoculated with AML1/ETO-positive Kasumi-1 cells (200×10^4^ cells/mouse) at the root of the right upper limb, and the pRNAi-siHO-1-K group was inoculated with pRNAi-siHO-1-GFP-transfected Kasumi-1 cells (200×10^4^ cells/mouse) at the root of the right upper limb.

### Changes after onset

Following the inoculation of each nude mouse group with Kasumi-1 cells, the body weight changes and the growth of subcutaneous nodules were observed and recorded. The survival times of the mice were evaluated by Kaplan-Meier survival curve.

### Routine blood testing

Blood was sampled (0.1–0.2 ml each time) from the distal end and then the proximal end of the tail vein by making a transverse incision with a disposable sterile scalpel blade. The blood was dropped into a tube containing ethylenediamine tetraacetic acid (EDTA) as an anticoagulant. Routine blood tests were performed to detect the changes of leukocyte and platelet counts as well as the hemoglobin levels.

### Detection of fusion gene AML1/ETO expression

Dying mice were killed by cervical dislocation that minimized pain and suffering. The ends of the femur were cut down, and bone marrow was collected. The liver, lung, spleen and kidneys of the mice were detached following the separation of the peritoneal cavity layer-by-layer. Total RNA was extracted from all the aforementioned organs that had been rinsed repeatedly with normal saline in order to detect the expression of AML1/ETO by qPCR. The method used TaqMan probes (Applied Biosystems) and an Eppendorf Sequence Detection System (Eppendorf, Hamberg, Germany). The probes and primers sequences used for AML1/ETO qPCR are as described in a Europe Against Cancer Program (18). AML1/ETO, forward: 5′-CACCTACCACAGAGCCATCAAA-3′, reverse: 5′-ATCCACAGGTGAGTCTGGCATT-3′ and probe: FAM-AACCTCGAAATCGTACTGAGAAGCACTCCA; ABL, forward: 5′-TGGAGATAACACTCTAAGCATAACTAAAGGT-3′, reverse: 5′-GATGTAGTTGCTTGGGACCCA-3′ and probe: FAM-CCATTTTTGGTTTGGGCTTCACACCATT. cDNA templates (2.5 μl) were added to each tube as with competitive PCR. Each qPCR assay was performed in a final volume of 25 μl under the following conditions: 95°C for 5 min, then 40 cycles at 95°C for 15 sec and 58°C for 1 min. The copy numbers of AML1/ETO were determined according to the standard curve.

### Statistical analysis

Data are expressed as mean ± standard deviation and analysis of variance (ANOVA) was performed with SPSS software, version 13.0 (SPSS Inc., Chicago, IL, USA). P<0.05 was considered as to indicate a statistically significant difference.

## Results

### Expression of HO-1 in AML-M2 patients

RT-PCR revealed that HO-1 was expressed at higher levels in the peripheral blood mononuclear cells of AML patients than in normal subjects (Fig. 1).

### HO-1 expression in BMMNCs

A lentiviral vector carrying HO-1 siRNA was constructed and used for the targeted silencing of HO-1 expression in BMMNCs. RNA and lysed proteins were extracted from the cells in the experimental groups that had been infected for 72 h. The relative expression levels of HO-1 mRNA and protein were confirmed to be reduced following targeted HO-1 silencing by qPCR and western blotting respectively (Fig. 2).

### Effects of targeted HO-1 silencing on survival rate

After 24, 48 and 72 h of treatment with DNR (0, 2.5, 5, 7.5, 10 and 12.5 μg/ml) respectively, the effects of HO-1 silencing on DNR-inhibited cell proliferation were determined by the CCK-8 method. As shown in Fig. 3, the survival rates of the BMMNCs correlated with DNR concentration in a time- and dose-dependent manner. After silencing with pRNAi-siHO-1-GFP, the survival rate of the cells clearly exceeded those of the BMMNC and pRNAi-GFP-BMMNC groups.

### Effects of HO-1 silencing on apoptotic rate

The cells treated with 5 and 10 μg/ml DNR for 48 h were collected and subjected to Annexin V-FITC and PI staining, and the apoptotic rates were measured by flow cytometry (Fig. 4). The apoptotic rate of the BMMNC group increased with rising DNR concentration. The apoptotic rates of the pRNAi-siHO-1-BMMNC group following treatment with 5 and 10 μg/ml DNR were 64.70±1.99 and 71.87±0.96% respectively, which were significantly higher than those of the BMMNC group (16.24±0.95 and 36.09±1.02%, respectively) and the pRNAi-GFP-BMMNC group (17.90±1.10 and 38.73±1.18%, respectively).

### mRNA expression of HO-1 and caspase-3, -8 and -9

To further explore the role of pRNAi-siHO-1-BMMNC in DNR-induced BMMNC apoptosis, the expression of caspase-3, -8 and -9 and HO-1 mRNA was detected by qPCR after 48 h of treatment with 0, 5, 7.5, 10 and 12.5 μg/ml DNR. Using GAPDH as the internal reference, relative expression levels were calculated by the 2^−ΔΔCt^ method and represented graphically. The expression level of HO-1 in the pRNAi-siHO-1-BMMNC group was lower than that in the BMMNC group (Fig. 5A), while those of apoptosis-related mRNAs increased (Fig. 5B–D). The expression levels of HO-1 and caspase-3, -8 and -9 mRNA increased as the concentration of DNR increased. Therefore, HO-1 siRNA may promote BMMNC apoptosis by a caspase activation cascade.

### Protein expression of HO-1 and caspase-3, -8 and -9

Lysed proteins were collected from the BMMNC group and the pRNAi-siHO-1-BMMNC group that had been treated with 5 μg/ml DNR. Using β-actin as the internal reference, the expression of HO-1 and apoptosis-related proteins was detected by western blotting. Following treatment with 5 μg/ml DNR, the expression level of HO-1 in the pRNAi-siHO-1-BMMNC group was lower than that in the BMMNC group, whereas those of the apoptosis-related proteins were higher (Fig. 6). Thus, the HO-1 siRNA-facilitated cell apoptosis was associated with the activation of caspases.

### Effects of HO-1 siRNA on the tumor formation outcomes of the established AML-M2 xenograft mouse model

The tumor formation outcomes and nodule volume changes of the four nude mouse groups are presented in Fig. 7A and B. No tumors formed in the blank or normal saline groups. Tumors formed in the Kasumi group on day 6 after inoculation when the nodules were ~0.4 cm in diameter, and the nodules further grew to ~1.7 cm on day 15. The pRNAi-siHO-1-K group developed tumors on day 10 after inoculation, with ~0.3-cm-diameter nodules that grew to ~1.2 cm on day 19. The body weight changes of the four groups are shown in Fig. 7C. The body weights of the blank and normal saline groups were almost unchanged. By contrast, the Kasumi group underwent a sharp reduction in body weight. The pRNAi-siHO-1-K group underwent a similar body weight reduction to that of the Kasumi group over a longer time period.

Blood samples were drawn from the tail veins of the four nude mouse groups on days 7, 14 and 21 after inoculation to determine the changes in the peripheral blood leukocyte and platelet counts as well as the hemoglobin levels. Compared with the blank and normal saline groups, the peripheral blood leukocyte and platelet counts and hemoglobin levels of the Kasumi and pRNAi-siHO-1-K groups were significantly reduced (P<0.05). The leukocyte counts were 9.25±0.76×10^9^/l on day 7 and 7.76±1.55×10^9^/l on day 14 in the Kasumi group, and 10.1±0.42×10^9^/l on day 7, 9.06±0.72×10^9^/l on day 14 and 7.22±0.76×10^9^/l on day 21 in the pRNAi-siHO-1-K group. The hemoglobin levels were 157.45±8.8 and 138.56±9.82 g/l in the Kasumi group on days 7 and 14, and 165.59±4.92, 159.06±6.86 and 147.22±10.5 g/l in the pRNAi-siHO-1-K group on days 7, 14 and 21, respectively. The platelet counts were 935.9±28.14×10^9^/l on day 7 and 618.4±129.89×10^9^/l on day 14 in the Kasumi group, and 985.8±16.92×10^9^/l on day 7, 798.5±86.54×10^9^/l on day 14 and 652.5±67.26×10^9^/l on day 21 in the pRNAi-siHO-1-K group. At each time point, the counts of leukocytes and platelets and hemoglobin level of the pRNAi-siHO-1-K group were significantly lower than those of the Kasumi group (P<0.05; Fig. 7D–F).

In Fig. 7G, the average survival times of the four nude mouse groups are shown to be 41.3±2.43, 40.2±5.56, 18.1±3.78 and 34.8±3.64 days in the blank, normal saline, Kasumi and pRNAi-siHO-1-K groups, respectively. Compared with the survival time of the Kasumi group, that of the pRNAi-siHO-1-K group was significantly extended (P<0.05).

### Expression of AML1/ETO

In order to assess the degree of infiltration of leukemic cells in different organs, the expression of AML1/ETO in the bone marrow, liver, spleen, lung and kidney was detected. As shown in Fig. 8, the copy numbers (x10^6^) of AML1/ETO fusion gene in the bone marrow, liver and spleen were 1.036±0.109, 0.230±0.456 and 0.160±0.033, respectively, in the Kasumi group and 0.333±0.195, 0.084±0.059 and 0.058±0.045, respectively, in the pRNAi-siHO-1-K group. The copy numbers in the lung and kidney were below the detection limit (1×10^3^). The expression level of AML1/ETO was increased in the bone marrow, liver and spleen in the Kasumi and pRNAi-siHO-1-K groups, indicating that the bone marrow, liver and spleen were subjected to diffuse filtration of leukemic cells. By contrast, the expression of AML1/ETO in the lung and kidney was undetectable, showing that the lungs and kidneys scarcely succumbed to infiltration by leukemic cells. The expression level of AML1/ETO in the Kasumi group was clearly higher than that in the pRNAi-siHO-1-K group.

## Discussion

HO-1 plays a vital role in tumorigenesis (19); HO-1 is generally highly expressed in tumor cells, which affects the response to treatment. Although the functions of HO-1 are tissue-specific, it is a key enzyme that contributes to the onset and development of tumors (20). In addition to heme, drugs as well as physiological and non-physiological stresses, for example, UV radiation, heat, inflammatory factors, microbial toxins and heavy metals, can induce the expression of HO-1 (21–25). The 5′-end of the HO-1 gene contains several binding sites for inflammatory and apoptotic transcription factors such as NF-κB, AP-1 and Nrf2 (24–26). Therefore, HO-1 expression is involved in cell biological processes through the regulation of transcription factors. Although HO-1 has been verified to exert anti-apoptotic effects on certain solid tumor cells (29), the impact of HO-1 expression in AML cells on biological processes remains to be elucidated.

In the present study, BMMNCs separated from AML-M2 patients were infected with a constructed lentivirus pRNAi-siHO-1-GFP to silence the expression of HO-1. qPCR and western blotting results demonstrated that the level of HO-1 expression in BMMNCs was significantly inhibited.

Subsequently, the effects of targeted HO-1 silencing on the apoptosis of BMMNCs induced by different concentrations of DNR were investigated. The survival rates of BMMNCs after 24, 48 and 72 h of treatment were detected by the CCK-8 method. The growth inhibition rate increased with rising DNR concentration and with extended treatment time. The group in which HO-1 expression was silenced had higher inhibition rates than the control and the blank vector groups did at each DNR concentration. Following treatment with 12.5 μg/ml DNR, the growth inhibition rates of the three cell groups gradually leveled off. Annexin V-FITC/PI double staining results demonstrated that the apoptotic rate of the pRNAi-siHO-1-BMMNC group was significantly higher than those of the other two groups, suggesting that targeted HO-1 silencing could raise the susceptibility of BMMNCs to DNR by enhancing the pro-apoptotic effects of DNR.

Given that HO-1 silencing inhibited cell survival and promoted apoptosis, the mRNA expression of apoptosis-related genes in the BMMNC and pRNAi-siHO-1-BMMNC groups that had been treated with series concentrations of DNR was detected by qPCR. With rising DNR concentration, the expression levels of caspase-3, -8 and -9 were elevated in a dose-dependent manner. Western blotting results revealed that the protein expression levels of apoptosis-related genes increased following treatment with 5 μg/ml DNR, particularly in the pRNAi-siHO-1-BMMNC group with targeted HO-1 silencing. Thus, targeted HO-1 expression is indicated to be conducive to the apoptosis of BMMNCs by facilitating the activation of these genes. Moreover, HO-1 expression in the pRNAi-siHO-1-BMMNC group was clearly suppressed, but remained dependent upon the concentration of DNR.

The anti-apoptotic and proliferation-inhibiting effects of targeted HO-1 silencing on AML cells were further elucidated *in vivo* by subcutaneously inoculating nude mice with AML1/ETO-positive Kasumi-1 cells.

The tumor formation outcomes, survival time and body weight changes of the mice were determined to clarify the routine test results of peripheral blood and to observe the infiltration of bone marrow, liver and spleen with grafted tumor cells. No tumors formed in the blank or normal saline groups, while all mice in the Kasumi and pRNAi-siHO-1-K groups developed tumors. They began to bear tumors on days 6 and 10, respectively, and the tumor size of the Kasumi group was significantly larger than that of the pRNAi-siHO-1-K group. Accordingly, HO-1 siRNA may inhibit the malignant proliferation of tumor cells, thus accelerating tumor growth to larger volumes. Kaplan-Meier survival curves demonstrated that the rats of the blank and normal saline groups survived longer, followed by the pRNAi-siHO-1-Kasumi group and the Kasumi group sequentially, indicating that HO-1 expression silencing was able to mitigate the filtration of tumor cells and to prolong the overall survival time. To detect the changes of leukocyte and platelet counts and hemoglobin levels, blood was collected at regular intervals. Since nude mice may die due to excessive bleeding or infections due to frequent sampling, blood samples were collected only on days 7, 14 and 21 after inoculation. Compared with the blank and normal saline groups, the leukocyte and platelet counts and hemoglobin levels of the two experimental groups, particularly those of the Kasumi group, decreased markedly. The results may be ascribed to the suppressed medullary hematopoiesis by the infiltration of Kasumi-1 cells. After blood sampling, the rats of the Kasumi and pRNAi-siHO-1-Kasumi groups did not stop bleeding immediately and required 2 min of local hemostasis, which can be attributed to the reduction of platelet count.

As evidenced by the expression of AML1/ETO, the bone marrow, liver and spleen of the rats of the Kasumi and pRNAi-siHO-1-Kasumi groups were infiltrated with leukemic cells, with those of the former group being more severe. Hence, HO-1 siRNA hindered the invasion of Kasumi-1 cells *in vivo*.

In short, targeted silencing of HO-1 expression was found to inhibit the proliferation of tumor cells, promote their apoptosis and relieve their infiltration into organs. The findings provide experimental evidence for the gene-targeted therapy of AML-M2. Nevertheless, the regulatory effects of HO-1 silencing on AML treatment in clinical practice require investigation in further studies.

In the present study, the *in vivo* and *in vitro* effects of targeted HO-1 silencing on the apoptosis of human M2-type leukemic cells were investigated. HO-1 silencing increased the susceptibility of BMMNCs to DNR and facilitated their apoptosis by caspase activation cascade. HO-1 silencing also suppressed the proliferation of solid tumor cells, enhanced their apoptosis and alleviated infiltration into organs. The results provide valuable evidence for the targeted therapy of M2-type leukemia. However, the detailed mechanisms for the role of downregulated HO-1 expression in the inhibition of tumor cell proliferation and promotion of apoptosis require elucidation by future in-depth studies.

## Figures and Tables

**Figure 1:** Expression of HO-1 mRNA in AML-M2 patients analyzed by reverse transcription-polymerase chain reaction. (A) HO-1 expression in the peripheral blood mononuclear cells of AML patients was detected by RT-PCR. (B) Relative expression of HO-1 shown in a bar chart using GAPDH as the internal reference. Patients 1–15, AML patients; Donors 1–15, normal subjects; M, marker; HO-1, heme oxygenase-1; AML, acute myelocytic leukemia.

**Figure 2:** Targeted silencing of HO-1 expression by pRNAi-siHO-1-GFP.(A) After 72 h of culture, significantly less HO-1 mRNA was expressed in the group infected with lentiviral vector carrying HO-1 siRNA than in the other two groups (P<0.05). (B) After 72 h of culture, western blotting results demonstrated that HO-1 protein expression in the pRNAi-siHO-1-BMMNC group was significantly downregulated (P<0.05). 1, BMMNC; 2. pRNAi-GFP-BMMNC; 3. pRNAi-siHO-1-BMMNC. HO-1, heme oxygenase-1; GFP, green fluorescent protein; siRNA, small interfering RNA; BMMNC, bone marrow mononuclear cell.

**Figure 3:** Inhibition of the survival of BMMNCs in various experimental groups by different concentrations of DNR analyzed by the CCK-8 method. Data are expressed as mean ± standard deviation based on the average of three repeated tests. After being treated with DNR for (A) 24, (B) 48 and (C) 72 h, respectively, the pRNAi-siHO-1-BMMNC group had significantly higher inhibitory rates than the other two groups did at each drug concentration and at each time interval (P<0.05). BMMNC, bone marrow mononuclear cell; DNR, daunorubicin; CCK-8, cell counting kit-8; GFP, green fluorescent protein.

**Figure 4:** Apoptotic rates of the three cell groups as detected by flow cytometry. (A) DNR induced cell apoptosis in a dose-dependent manner. Following treatment with 5 and 10 μg/ml DNR for 48 h, the apoptotic rates of the pRNAi-siHO-1-BMMNC group were significantly higher than those of the other two groups (P<0.05). (B) Apoptotic rates obtained from three repeated experiments (mean ± standard deviation). DNR, daunorubicin; BMMNC, bone marrow mononuclear cell; GFP, green fluorescent protein; HO-1, hemo oxygenase-1.

**Figure 5:** HO-1 and caspase-3, -8 and -9 mRNA expression was detected by quantitative polymerase chain reaction. (A) HO-1 mRNA expression changed depending on the dose of DNR. The expression level increased with rising DNR concentration and peaked in the presence of 10 μg/ml DNR. Expression levels of (B) caspase-3, (C) caspase-8 and (D) caspase-9 mRNA in the pRNAi-siHO-1-BMMNC group were higher than those in the BMMNC (control) group at each DNR concentration, the differences in the mRNA expression levels above were statistically significant (P<0.05). Expression levels increased with rising DNR concentration and peaked in the presence of 10 μg/ml DNR. HO-1, heme oxygenase-1; DNR, daunorubicin; BMMNC, bone marrow mononuclear cell.

**Figure 6:** Expression of HO-1 and caspase-3, -8 and -9 proteins. Following treatment with 5 μg/ml DNR, the expression levels of caspase-3, -8 and -9 proteins in the pRNAi-siHO-1-BMMNC group were higher than those in the BMMNC group, whereas HO-1 protein expression was silenced. The differences in protein expression were statistically significant (P<0.05). HO-1, heme oxygenase-1; DNR, daunorubicin; BMMC, bone marrow mononuclear cell.

**Figure 7:** Changes of body weight, leukocyte and platelet counts and hemoglobin levels, and Kaplan-Meier survival curve in the nude mouse model. (A) The Kasumi-1 cell-inoculated nude mouse model; left, Kasumi group; right, pRNAi-siHO-1-K group. (B) Volume of subcutaneous nodules in the nude mouse model; left, Kasumi group; right, pRNAi-siHO-1-K group. (C) Body weight changes of the blank, normal saline, Kasumi and pRNAi-siHO-1-Kasumi groups were recorded every 5 days. The body weights of the Kasumi group and the pRNAi-siHO-1-K group decreased from day 5, and that of the Kasumi group dropped to a greater extent. (D) Changes of leukocyte counts. The count of the Kasumi group reduced significantly (P<0.05). (E) Changes of hemoglobin levels. The hemoglobin level in the peripheral blood of the Kasumi group was significantly reduced (P<0.05). (F) Changes of platelet counts. The count of the Kasumi group was significantly lower than those of the other three groups (P<0.05). (G) Kaplan-Meier survival curves for evaluating the survival time of nude mice. The pRNAi-siHO-1-K group survived longer than the Kasumi group did. WBC, white blood cell; PLT, platelet; Hb, hemoglobin; HO-1, heme oxygenase-1.

**Figure 8:** Copy number of AML1/ETO fusion gene as detected by quantitative polymerase chain reaction. AML1/ETO expression in the bone marrow, liver and spleen was significantly higher than that in the lung and kidney. In the Kasumi group, the expression of AML1/ETO was higher than that in the pRNAi-siHO-1-K group. HO-1, heme oxygenase-1.

**Table I:** Primer sequences of HO-1^RT^, HO-1, caspase-3, caspase-8, caspase-9 and GAPDH genes.

Gene	Forward	Reverse	Product (bp)
HO-1^RT^	5′-GCAGTCAGGCAGAGGGTGATAGAAGAGG-3′	5′-CTGAGTGTAAGGACCCATCGGAGAAGC-3′	305
HO-1	5′-AGCTTGGTCTAGAGTGAAAA-3′	5′-GAGGCAGAATCATGAGATAT-3′	180
Caspase-3	5′-GACTCTGGAATATCCCTGGACAACA-3′	5′-AGGTTTGCTGCATCGACATCTG-3′	140
Caspase-8	5′-CAAGAGGAAATCTCCAAATGCAAC-3′	5′-CAGGATGTCCAACTTTCCTTCTCC-3′	108
Caspase-9	5′-GAGCAGTGGGCTCACTCTGAA-3′	5′-GGAAATTAAAGCAACCAGGCATC-3′	106
GAPDH	5′-GAAGGTGAAGGTCGGATGC	5′-GAAGATGGTGATGGGATTTC	226

HO-1, heme oxygenase-1 for quantitative polymerase chain reaction; HO-1^RT^, heme oxygenase-1 for reverse transcription polymerase chain reaction.
